RETRACTED

# Early Assessment of Cardiac Function by Echocardiography in Patients with Gestational Diabetes Mellitus

**DOI:** 10.1155/2022/6565109

**Published:** 2022-08-27

**Authors:** Pin Wang, Yanyan Peng, LiNa Liu, RuiShuang Jiao, YanHong Zhang, Wei Zhao, YingFeng Liu, CongXin Sun

**Affiliations:** ^1^Shijiazhuang Obstetrics and Gynecology Hospital Ultrasonography Lab, 050000, China; ^2^Gucheng County Hospital of Hebei Province Obstetrics and Gynecology Ultrasound Department, 253800, China; ^3^The Third Hospital of Shijiazhuang Ultrasonography Lab, 050000, China

## Abstract

**Objective:**

To offer a baseline for clinical diagnosis, echocardiography was performed to evaluate the disparities in heart function comparing pregnant women with diabetes mellitus (GDM) and ordinary pregnant women.

**Methods:**

A prospective case-control study is being conducted on pregnant women with or without gestational diabetes. The sample size for both the intervention and control groups is the same: no diabetes diagnosis or previous forms, a single pregnancy, and no issues (such as preeclampsia or fetal growth restriction). The females were all subjected to routine echocardiograms to examine the morphology and function of their left and right hearts.

**Results:**

In the research, 51 women with GDM and 50 healthy controls volunteered. Women with GDM had a significantly higher heartrate (82 ± 9 vs. 74 ± 8), left ventricular (LV) relative wall thickness (0.39 ± 0.06 vs. 0.31 ± 0.07; *P* < 0.001), LV early diastolic transmitral valve velocity (E) (0.79 ± 0.14 vs. 0.72 ± 0.13 m/s; *P* = 0.031), and LV late diastolic implementing regulations valve velocity (0.6). Speckle-tracking analysis showed significant decrease in LV right ventricular (RV). A study indicated a reduced pulmonary acceleration time (59 ± 9 vs. 68 ± 12 ms; *P* = 0.001), RV E/A ratio (1.21 ± 0.19 vs. 1.31 ± 0.31; *P* = 0.022), and a greater RV myocardial systolic annular velocity (0.17 ± 0.03 vs. 0.12 ± 0.03; *P* = 0.023).

**Conclusions:**

Our results revealed that the heart function of diabetic pregnant women differed considerably from that of the control group, such as LV-RWT, LV diastolic transmitral valve speed, and LV late diastolic transmitral valve speed. Given these results, further research into the postpartum cardiovascular healing of pregnant women with gestational diabetes mellitus is required.

## 1. Introduction

Gestational diabetes (GDM) refers to women who have no symptoms of diabetes before and have symptoms of hyperglycemia during pregnancy [1]. Gestational diabetes may not have obvious symptoms, but it will increase the risk of pregnancy toxemia and depression and the possibility of cesarean section [2]. If a pregnant woman has gestational diabetes and is not properly treated, it may increase the risk of infant overgrowth, postnatal hypoglycemia, or jaundice [3]. In serious cases, it may also cause stillbirth, and the risk of childhood obesity and type 2 diabetes after children grow up is relatively high [4]. Hyperglycemia during pregnancy can lead to abnormal embryonic development and even death, and the incidence of abortion is 15%-30%. The probability of pregnancy-induced hypertension is 2-4 times higher than that of nondiabetes pregnant women [5]. The incidence of polyhydramnios was 10 times higher than that of nondiabetes pregnant women. The incidence of macrosomia is significantly increased, the probability of dystocia, birth canal injury, and surgical delivery is increased, and the labor process is prolonged, which is prone to postpartum hemorrhage [6]. In addition, it is prone to diabetes ketoacidosis and infection related to gestational diabetes, such as vulvovaginal candidiasis, pyelonephritis, asymptomatic bacteriuria, puerperal infection, and mastitis [7]. If pregnant women with diabetes do not receive timely and effective treatment and management, their future risk of type 2 diabetes will increase. At the same time, pregnant women with diabetes also have a higher risk of preeclampsia and cesarean section [8].

RETRACTED

Previous research has shown that gestational diabetes mellitus has an influence on the heart, and in more severe situations, it may even lead to malfunction [9]. This malfunction may express itself in a number of ways, including cardiomyopathy, microvascular protrusions, and subcellular issues [10]. Patients with type 2 diabetes suffer from both structural and functional heart damage as a result of these complications. On either hand, scientists know a little about the implications of hyperglycemia, which for a short period of time, on the hearts of patients who have gestational diabetes [11]. There have been no prospective studies to look at how gestational diabetes impacts the mother's cardiac function. The goal of this study was to compare and contrast the cardiac function of pregnant women who had or did not have diabetes. [12]. Our working hypothesis was gestational diabetes can affect the cardiac function and structure of pregnant women.

## 2. Material and Methods

### 2.1. Selection of Subjects

Our hospital will conduct a 12-month prospective study from July 2019 to July 2020. The hospital's Ethics Review Committee (12/L1/2019) approved and carried out the study, and written informed consent was obtained from all pregnant women and their families. An oral glucose tolerance test was used to diagnose GDM in these pregnant women at 20 and 2 weeks.  Figure 1 shows ultrasound images of both normal and pregnant women.

RETRACTED

### 2.2. Glucose Tolerance Experiments

Glucose tolerance tests are one method for investigating human blood glucose regulating systems. Subjects were given a single oral dose of 75 g of glucose dissolved in 250 mL of warm boiled water within 5 minutes of drinking completely, venous blood was drawn at each of the three time points (1 hour, 2 hours, and 3 hours), and urine samples were retained after each blood draw for determination of blood glucose and urinary glucose. At the time of fasting, the blood glucose level in normal people is in the range of 3.9-6.1 mmol/L; after 1 hour of oral administration of glucose, the blood glucose concentration reaches a peak, usually in the range of 7.8-9.0 mmol/L; the peak value does not exceed 11.1 mmol/L; the 2-hour blood glucose is less than 7.8 mmol/L; and the blood glucose returns to the fasting level after 3 hours. Urine sugar levels were negative at all testing times. However, diabetic patients' fasting blood glucose levels were often higher than 7.0 mmol/L, their OGTT peak blood glucose level was higher than 11.1 mmol/L, and their 2-hour blood glucose level was similarly higher than 11.1 mmol/L, accompanied by positive urine glucose.

### 2.3. Inclusion Criteria

There were no prior diabetes or cardiovascular problems (type 1 or 2). Body mass index (BMI) of healthy pregnant women was 30 kg/m^2^ with no comorbidities. The pregnant women included in the study had normal blood pressure, single pregnancy, normal fetal development, and no preeclampsia symptoms.

### 2.4. Echocardiographic Examination

A senior professional examiner evaluated and analyzed the hearts of pregnant women using a Siemens 4v1c color Doppler ultrasonography diagnostic device (ACUSON oxana2). The patient was in the left decubitus position, and the image was detected by sternum and apical angle. Use the hard disk to copy all the data of three heart cycles in the ultrasound instrument and follow-up analysis. The investigation was designed to comply with the most recent standards. Samples were recorded of the left atrial volume (LAVI), the close volume of the left ventricle (LV), the radii of the distal (RD), and proximal RV outflow systems, and other geometric indices(GI) using dorsal long-axis (DLA), quick, and apex five views. The early (E) and late (A) mitral and tricuspid ventricular inflow velocities (IV), acceleration time (T), isovolumetric relaxation (IR), and late mitral leaflet inflow duration may also be determined using dynamic imaging. Tissue with pulsed pulses Doppler imaging is also used to determine the systolic (S), early-diastolic (E), and latdiastolic (A) velocities of heart tissue so at septum, “L”, and “RV” walls. “LVM” was determined by applying the following formula, which was derived from the “Essex equation”: (LVM) = 0.8 (1.04((LVEDD + IVSd + PWd)3–LVEDD 3) + 0.6, in which LVEDD is the LV end-diastolic diameter, IVSd is the ventricular septal defect thickness in the diastole, and “PWd” is the posterior wall thickness in the diastole. The LV mass index (LVMI) was calculated by taking the LVM and dividing it by the total surface area of the body. RWT = (2 PWd)/LVEDD was the formula that was used to determine the LV ratio wall thickness (RWT). The recommendations provided by the British Society of Echocardiography were utilized in order to diagnose diastolic dysfunction. These recommendations used values that were adjusted for age and gender and were taken from the 2016 European Society of Cardiology Guidelines for the Diagnosis and Management of Acute and Chronic Heart Failure. Calculations were done based on the apical pictures to determine the LV and RV global longitudinal strain (GLS), as well as the systolic and diastolic (early and late) strain rates. Negative values indicated that the fibers were being shortened. Apical and basal parasternal short-axis photos were utilized to determine LV rotation and derotation, with negative values indicating rotation clockwise. The LV twist distinguishes between the apical and basal rotations of the rotors. To determine LV torsion, divide the LV twist by the diastole length of the LV. There was no statistical analysis for those who refused to participate in more than one section.

RETRACTED

### 2.5. Statistical Analysis

The mean standard deviation of continuous data is shown. The Shapiro–Wilk test is used to test normal distribution. The chi-square test was used to compare categorical data that was given as *n*. (percentages). In order to do group comparisons, we either used the unpaired *t*-test or the Mann–Whitney *U*-test with continuous data. The choice of which test to use was dependent on the distribution of the data. The significance level was set at *P* < 0.05. IBM SPSS software version 24 was used for statistical analysis (IBM Corp., Armonk, NY, USA). Previously, our team discovered intra- and interobserver heterogeneity, which was not repeated in our investigation.

## 3. Results

### 3.1. Conditions of Participating Study Patients

This research included 101 pregnant women, 51 of whom had gestational diabetes and 50 who were healthy (control group). All of the ladies underwent routine echocardiogram satisfactorily.  Figure 2 depicts the demographic features of the control group and women with gestational diabetes. When compared to controls, women with gestational diabetes had substantially higher BMI and systolic blood pressure.

RETRACTED

### 3.2. Comparison of Ultrasound Parameters

Figure 3 shows the echocardiographic indices for both groups. There was no statistical significance to the difference. When compared to the controls, the GDM women had significantly greater levels of physical activity, LV-RWT, LV diastolic transmitral valve speed, and LV late diastolic transmitral valve speed. Keeping in mind that the LVM and LVMI did not vary at all between the two groups is critical, since this is a crucial point to remember. When compared to control pregnancies, a chronic strain assessment of the LV showed that global longitudinal strain (GLS), endocardial GLS, and dural GLS all decreased by a lot. This was proven by comparing pregnancies with GDM to those without it. When compared to the control group, women with GDM had a shorter pulmonary acceleration time, a lower RV E/A ratio, and larger RV-S and RV-A values. Also, the RV-S and RV-A values were higher for these women. Speckle-tracking was used to look at the right ventricle, and the results showed that there were no big differences between the women with GDM and the controls (Figures 4–9).

## 4. Discussion

Patients with gestational diabetes exhibited substantially higher LV-RWT and lower LV-GLS, LV endocardial, and epicardial GLS compared to the control group, according to echocardiographic data [13]. As a result, women with gestational diabetes had significantly worse heart function throughout pregnancy when compared to the healthy control group [14]. Despite the absence of clinical symptoms in these individuals, this clear cardiovascular adverse response may offer a concern to pregnant women [15]. Previously, researchers employed the speckle tracking technology to examine the systolic function of diabetic patients with normal blood pressure and discovered that GLS and endocardial hypotension of the left ventricle were decreased [16]. However, the cardiovascular effects of diabetes may be mistaken with metabolic syndrome, which includes hypertension and dyslipidemia in addition to high blood glucose levels [17]. The longitudinal and circumferential strains of lv22 and 23 reduced, as did the GLS of rv24, in a study of cardiac alterations in metabolic syndrome [18]. Short-term hyperglycemia during pregnancy has the same effect on heart function as non-pregnant people with a long history of diabetes. Researchers discovered that the GLS of radial strain differed in a retrospective analysis of 18 pregnant women with gestational diabetes in the second trimester of pregnancy [19]. Although the data in this section of the research are comparable to the findings in this study, it cannot be ruled out that these cardiovascular abnormalities are due to the small sample size, early gestational weeks at the time of examination, and brief exposure to hyperglycemia [20].

RETRACTED

Recent research has shown that hypertensive disorders of pregnancy and fetal development are linked to major problems with how the heart works in women [21]. GDM is a major risk factor for many diseases [22]. Someone is more likely to get GDM if they have GDM. We may have contributed to exclusion bias by not checking on women who had heart problems because of these pregnancy problems and by leaving out women with GDM who had these worries from a prospective study [23]. According to our data, this means that, unlike when PE or FGR start, when the heart function gets worse, the heart function is normal during a GDM pregnancy [24]. Despite these problems, women with GDM are about 2.8 times more likely to have diastolic dysfunction than women who have a normal pregnancy to term. Researchers have found that this link makes it more likely for pregnant women to get heart disease [25]. We do not fully understand how diabetes can change the rhythm of the heart in nonpregnant people. Diabetic cardiomyopathy includes a wide range of problems, such as myocardial fibrosis and remodeling, problems with the heart's ability to pump blood, and problems with the heart's ability to pump blood at all. It is usually called diabetic cardiomyopathy. Diabetes has been linked to inflammation, activation of the renin-angiotensin-aldosterone system, microvascular dysfunction, and bad insulin signaling in the heart. Also, people with diabetes are more likely to develop type 2 diabetes [26].

A new meta-analysis shows that women who develop impaired glucose tolerance during pregnancy are 1.5 times more likely to have a heart attack in the first year after giving birth. This higher risk exists whether or not the woman develops type 2 diabetes after giving birth [26]. The authors thought that both GDM and PE might make pregnant women more likely to have heart problems after giving birth. It is interesting to think about how the pathophysiology of GDM fetal circulatory failure could lead to long-term heart damage and fibrosis, like what happens in diabetic cardiomyopathy [27]. Future research should focus on how the heart works after giving birth to a baby with gestational diabetes mellitus. This will help find out if this problem is just caused by the GDM pregnancy or if it is hidden by the effects of other heart risk factors [28]. One of the study's strengths is that it was set up in a prospective way and used both traditional and speckle-tracking sonar to measure how well the left and right hearts worked. A problem with the research is that the women with GDM at the start of the trial had a higher BMI and systolic blood pressure. It is impossible to say how much each of the above factors played a role in the development of heart problems during a GDM pregnancy [29]. In our study, heart problems were seen in mothers who did not have diabetes if their BMI was more than 35 kg/m^2^. This was a lot higher than the BMI of our GDM sample. Compared to pregnant women with BMIs less than 35 kg/m^2^, those with BMIs more than 35 kg/m^2^ had much higher SV, CO, and LVM, as well as much lower overall vascular resistance (TVR) [30].

RETRACTED

Except for LVMI, all of the differences went away when the weight of the mother was taken into account. In terms of SV, SV index, CO, CI, LVM, LVMI, TVR, and the receipt of the notice index, there was no difference between the GDM group and the controls [31]. So, we know for sure that the difference in speckle tracking and diastolic dysfunction is caused by GDM and not by the higher BMI reported in the GDM group. Surprisingly, it was found that pregnant women with gestational diabetes had more diastolic dysfunction than pregnant women who were obese. Also, women with GDM had their scans done two weeks before women in the control group. Because of the way the mother's heart changes during pregnancy, the second difference would have tended to reduce any differences between GDM and normal pregnancy rather than make them bigger.

## 5. Conclusions

The occurrence of short-term hyperglycemia in pregnant women with gestational diabetes may have a certain impact on cardiac function. Pregnant women with gestational diabetes have an increased risk of cardiovascular disease after delivery, so it is necessary to take preventive measures for such patients.

## Figures and Tables

**Figure 1:** Ultrasonogram of normal and pregnant women.

**Figure 2:** Demographic features of all participating pregnant women.

**Figure 3:** Ultrasonic parameter used in the study.

**Figure 4:** Tricuspid inflow index comparison.

**Figure 5:** Compare of strain and SR indices.

**Figure 6:** Hemodynamic index comparison.

**Figure 7:** Geometric index comparison.

**Figure 8:** Mitral inflow indices.

**Figure 9:** Strain and SR indices part II.

## Data Availability

All of the data in this article are actually available.
